The article "The Application of Wavelet-Domain Hidden Markov Tree Model in Diabetic Retinal Image Denoising" was published in 2015. Journal: Open Biomed Eng J.

# The Application of Wavelet-Domain Hidden Markov Tree Model in Diabetic Retinal Image Denoising

**DOI:** 10.2174/1874120701509010194

**Published:** 2015-08-31

**Authors:** Dong Cui, Minmin Liu, Lei Hu, Keju Liu, Yongxin Guo, Qing Jiao

**Affiliations:** 1 Department of Radiology, Taishan Medical University, Taian 271016, P.R. China; 2 Ophthalmology, Hospital of Traditional Chinese Medicine, Taian 271000, P.R. China; 3 Ophthalmology, Hospital Affiliated to Taishan Medical University, Taian 271000, P.R. China

**Keywords:** Fundus images, HIDDEN Markov Tree Model (HMT Model), image denoising, wavelet transform

## Abstract

The wavelet-domain Hidden Markov Tree Model can properly describe the dependence and correlation of fundus angiographic images’ wavelet coefficients among scales. Based on the construction of the fundus angiographic images Hidden Markov Tree Models and Gaussian Mixture Models, this paper applied expectation-maximum algorithm to estimate the wavelet coefficients of original fundus angiographic images and the Bayesian estimation to achieve the goal of fundus angiographic images denoising. As is shown in the experimental result, compared with the other algorithms as mean filter and median filter, this method effectively improved the peak signal to noise ratio of fundus angiographic images after denoising and preserved the details of vascular edge in fundus angiographic images.

## 1 INTRODUCTION 

As the incidence of diabetes has steadily increased in recent years, there are more and more patients of diabetic retinopathy (DR). DR as one of the most serious complications of diabetes, is one of the major cause of blindness currently, which has the concealed feature and the feature of irreversibility. Fluorescein fundus angiography (FFA) has an instructive significance on the early diagnosis and timely treatment of the DR [1-4]. In the collecting process of fundus angiographic images, factors like the nonuniformity of light, the imaging effect of fundus camera and the severe interference of noise in imaging process, such as the internal noise of sensitive components, optical material grain noise, thermal noise, transmission channel interference, quantization noise. Caused problems like the declined contrast ratio of fundus angiographic images, the severe interference of noise and image blurring, which influenced the clinical diagnosis of doctors. Therefore, the denoising of fundus angiographic images has important practically value in clinical appliance. Traditional image denoising methods, such as the median filter and the threshold algorithm, would lose quiet a little high frequency information in denoising, which caused the edge blur of images and the missing of detailed information [5-7]. Wavelet transform in the time domain and frequency domain also has good localization properties, Not only will the image structure and texture are represented in different resolution levels, but also has the ability to detect edge, wavelet transform could properly maintain the edge and features of details for imagesat the same time of denoising [8, 9]. Donoho [10] first proposed the wavelet shrinkage method, presented a method to calculate the universal threshold, proved the asymptotic optimality of general threshold, but the universal threshold used by the method has the tendency of excessive killing of wavelet coefficients. The literature [11]through the establishment of wavelet coefficients Gaussian mixture model, in order to maximize access to images of a priori information to improve the performance of denoising. Crouse [12]analyzed the wavelet coefficients of clustering and persistence, the wavelet coefficients proposed by hidden Markov tree (HMT) and Gaussian mixture model, and the model is used for one-dimensional signal denoising and classification. Because HMT model can well describe the correlation among wavelet coefficients and the maximum description image prior information, so it can be to remove the image noise, also to maintain a good image edge and details at the same time, the performance s(t) improvement of wavelet denoising algorithm. In this paper the wavelet-domain HMT was applied to describe the images and calculate the correlation of wavelet coefficients in neighbor scales [13], and an Bayesian estimation was implemented to estimate image models, which can help to properly maintain the edge information for images in the process of effective fundus angiographic images denoising. As the experimental result showed, the peak signal noise ratio (PSNR) and the visual quality of FFA denoising images were obviously improved.

The article "The Application of Wavelet-Domain Hidden Markov Tree Model in Diabetic Retinal Image Denoising" was published in 2015. Journal: Open Biomed Eng J.

## 2. THE WAVELET TRANSFORM

The wavelet transform refers to the signal expressed with the scaling and translation of wavelet function and scaling function [14]. 

The wavelet transform refers to the signal expressed with the scaling and translation of wavelet function ϕ(t)  and scaling function Φ(t) [14].

(1) $$\phi_{J,K}\left(t\right)=2^{-J/2}\phi \left(2^{-J}t-K\right)$$

(2) $$\Phi_{J,K}\left(t\right)=2^{-J/2}\Phi \left(2^{-J}t-K\right)J,K\in Z$$

The signal s(t)  can be expressed as:

(3) $$s\left(t\right)=\sum_{K}\mu_{K}\Phi_{J_{0},K}\left(t\right)+\sum_{J_{1}}^{J_{0}}\sum_{K}\omega_{J,K}\phi_{J,K}\left(t\right)$$

In the formula (3):

(4) $$\mu_{K}=\int s\left(t\right)\Phi_{J_{0},K}^{*}\left(t\right)dt$$

(5) $$\omega_{J,K}=\int s\left(t\right)\phi_{J,K}^{*}\left(t\right)dt$$

In the formula (3): J is the scale, J smaller the higher the resolution, K is the translation factor. In the practical application, resolution of s(t)  is limited. The scope of J is: $J\in \left[J_{1},J_{0}\right],J_{1},J_{0}\in Z$ .

Fast algorithm of wavelet decomposition can use the tower algorithm, Two-dimensional wavelet transform can be respectively to one dimensional wavelet transform rows and columns. Fig. (**1**) shows the various permutations of the different sub-bands of wavelet coefficients, L and H respectively expressed low-pass filter and high-pass filter. In addition to the scale biggest and smallest scale, under this kind of organization, each wavelet coefficients have four child nodes, a parent node. As shown in Fig. (**1**).

## 3 THE WAVELET-DOMAIN HMT MODEL

The energy compactness of wavelet transform shows, most change of images are composed by many small coefficients and a few large coefficients. The number set of large coefficients is the product of probability density function with large variance, while the number set of small coefficients is the product of probability density function with small variance. Thus, the Probability Density Function $f_{W}\left(w_{i}\right)$  of every wavelet coefficient w_i_could be well approximated by Gauss Mixture Model with dual density[14,15].

Supposing the Discrete Hidden State S_i_ of every wavelet coefficient w_i_is valued as m = S and L , and there is Probability Density Function $p_{S_{i}}\left(m\right)$ . Among which, S is the corresponding Gauss state of zero mean and small variance $\sigma_{S}^{2}$ , and L is the corresponding Gauss state of zero mean and large variance $\sigma_{L}^{2}and\sigma_{L}^{2}>\sigma_{S}^{2}$ .

Let

(6) $$g\left(x;u,\sigma^{2}\right)=\frac{1}{\sigma \sqrt{2\pi }}\exp\left\{-\frac{{\left(x-u\right)}^{2}}{2\sigma^{2}}\right\}$$

is the Gauss probability density function, then

(7) $$f_{W}\left(w_{i}|S_{i}=S\right)=g\left(w_{i};0,\sigma_{S;i}^{2}\right)$$

(8) $$f_{W}\left(w_{i}|S_{i}=L\right)=g\left(w_{i};0,\sigma_{L;i}^{2}\right)$$

the edge probability density function of wavelet coefficient w_i_ can be shown as:

(9) fW(wi)=piSg(wi;0,σS;i2)+piLg(wi;0,σL;i2) and piL+piS=1

The HMT Model of the image is quadtree structures [16], as is shown in Fig. (**2**). Each black node stands for a wavelet coefficient, and the white circle connected with the black node stands for the corresponding hidden state, by both of which a node is composed. The relation between Node 1 and Node 2-5 is the relation between parent nodes and child nodes, and so as the relation between Node 2 and Node 6-9. The link between Node 1 and Node 2 reflects the correlation across scales between Wavelet Coefficient 1 and Wavelet Coefficient 2, and the link between Node 2-5 and Node 1 reflects the correlation inside scales among Wavelet Coefficient 2-5. The size of wavelet coefficients is greatly connected with the parent node. Let the Hidden Status $\left\{S_{\rho \left(i\right)},S_{i}\right\}$  be a parent-child pair, ρ(i)  be the parent node of Node i, and $p_{i,m}^{\rho \left(i\right),m}$  be the state transition probability from State m to State $m^{\prime }$ , then the corresponding state transition matrix is:

(10) $$A_{i}=(\begin{array}{l} p_{i,S}^{\rho \left(i\right),S}\\ p_{i,S}^{\rho \left(i\right),L} \end{array}\begin{array}{l} p_{i,L}^{\rho \left(i\right),S}\\ p_{i,L}^{\rho \left(i\right),L} \end{array})=(\begin{array}{l} p_{i,S}^{\rho \left(i\right),S}\\ 1-p_{i,L}^{\rho \left(i\right),L} \end{array}\begin{array}{l} 1-p_{i,s}^{\rho \left(i\right),S}\\ p_{i,L}^{\rho \left(i\right),L} \end{array})$$

Therefore, the two dimensional HMT Model can be characterized through the mixture of $\sigma_{S;i}^{2}and\sigma_{L;i}^{2}$ , the State Transition Matrix A_i_, the every _i_ corresponding to every scale, and the probability $p_{i}^{L}$  which keeps in a large state in root node.

The article "The Application of Wavelet-Domain Hidden Markov Tree Model in Diabetic Retinal Image Denoising" was published in 2015. Journal: Open Biomed Eng J.

The HMT Model under the State M could be parameterized through the Probability Quality Function $p_{S_{i}}\left(m\right)$  of Node S_i_, the conditional probability $\varepsilon_{i,\rho \left(i\right)}^{m,r}$  of giving State $S_{\rho \left(i\right)}$  under the State r, that of S_i_ under the State m, and the Mean Value $\mu_{i,m}$ and the Variance $\sigma_{i,m}^{2}$  of Wavelet Coefficient W_i_ supposing the giving state $S_{\rho \left(i\right)}$  was under the State m.

All these parameters can be grouped into a parameter vector

(11) $$\vartheta =\left\{p_{S_{i}}\left(m\right),\varepsilon_{i,\rho \left(i\right)}^{m,r},\mu_{i,m},\sigma_{i,m}^{2}|i=1,2\cdots ,P;n,m=1\cdots M\right\}$$

Among which, P is the number of nodes; M is the state number.

## 4 THE REALIZATION OF HMT ALGORITHM

In HMT Model, State S_i_ is hidden and the expectation maximization(EM) algorithm is usually adopted to the observable wavelet coefficients. EM Algorithm is a kind of iterative algorithm, which can not only estimate the parameter vector but also the probability of the Hidden State S_i_[15, 17].

### 4.1 Model Training

Given a set or more sets of observed wavelet coefficients $w=\{w_{1},w_{2},\cdots ,w_{n}\}$ , can determine the best features of the wavelet coefficients of the wavelet-domain HMT parameter vector ϑ. Expectation maximization algorithm observed the wavelet coefficients w, can be estimate model parameters vector ϑ and the probability of hidden state S. The EM algorithm for HMT iterative format as follows.

The article "The Application of Wavelet-Domain Hidden Markov Tree Model in Diabetic Retinal Image Denoising" was published in 2015. Journal: Open Biomed Eng J.

Choose an initial model to estimate ϑ_0_ and let the iterative order l = 0, and then

⊝ Step E, to calculate the joint probability density quality function $p\left(S|w,\vartheta^{l}\right)$  of hidden state variable;

⊜ Step M, to calculate the new model parameter

$\vartheta^{l+1}=\arg\underset{\vartheta }{\max}E_{S}\left[\ln f\left(w,S|\vartheta \right)|w,\vartheta^{l}\right]$ ;

⊛ If $\vartheta^{l}=\vartheta^{l+1}$ , stop; otherwise, let l=l+1  and go back to Step E.

M step includes wavelet coefficients as a function upgrade of the mean , variance, transition probabilities, edge state probability mass function $p\left(S_{i}=m|w,\vartheta^{l}\right)$ , and parent-child probability mass function $p\left(S_{i}=m|w,S_{\rho (i)}=n,\vartheta^{l}\right)$ .

E steps to calculate these functions.

### 4.2 Likelihood Determination

Giving the wavelet domain HMT of Vector Parameter ϑ, and confirm the observation of Likelihood f(w|ϑ)  of Wavelet Coefficient w.

### 4.3 State Estimation

Giving the wavelet domain HMT with vectors, and for the observed Wavelet Coefficient $\left\{w_{i}\right\}$ , confirm the most possible sequence of Hidden State $\left\{S_{i}\right\}$  and the probability of Node i under a certain state.

## 5 THE BAYESIAN ESTIMATION OF IMAGE WAVELET COEFFICIENT 

Under the Gauss noise with the mean value of 0 and the variance of, the size of the image is, and N is the integer power of two. After the wavelet transform of images with Scale, we gained the Tree of wavelet coefficient with noise [15, 16, 18]. Then the relation among the Wavelet Coefficient of images with noise, the Wavelet Coefficient of original images and the Wavelet Coefficient of noises can be shown in wavelet domain as:

(12) $$w_{i}=y_{i}+n_{i}$$

Use the EM algorithm, fit a HMT model of y_i_ in the observed data w_i_, If the signal has a HMT probability density function of wavelet domain, then the signal containing noise also has a probability density function. Increase zero-mean independent Gaussian white noise n_i_, Each mixture model variance $\sigma_{i,m}^{2}$  increased by $\sigma_{n}^{2}$  and other parameters remain unchanged. Through the wavelet coefficient fitted the observed data of HMT minus the variance due to added noise, get the signal wavelet coefficients model.

Supposing in Scale L , the distribution of all state variables and wavelet coefficients were the same and so as the state transition matrix of parent and child nodes. Then under the condition that the State S_ i_ of Wavelet Coefficient y_i_ had been known, the conditional mean value could be estimated as:

(13) $$E\left[y_{i}|w=w_{i},S_{i}=m\right]=\frac{\sigma_{i,m}^{2}}{\sigma_{n}^{2}+\sigma_{i,m}^{2}}w_{i}$$

Supposing the wavelet coefficient and the model had been known, Hidden Probability $p\left(S_{i}|w,\vartheta \right)$  could be produced. With these state probability, the conditional mean estimation of y_ i_can be gained as

(14) $$E\left[y_{i}|w,\vartheta \right]=\sum_{m}p\left(S_{i}=m|w,\vartheta \right)\frac{\sigma_{i,m}^{2}}{\sigma_{n}^{2}+\sigma_{i,m}^{2}}w_{i}$$

Finally, the denoised images can be completed by inverse wavelet.

The article "The Application of Wavelet-Domain Hidden Markov Tree Model in Diabetic Retinal Image Denoising" was published in 2015. Journal: Open Biomed Eng J.

## 6 THE RESULT AND CONCLUSION OF EXPERIMENT 

The experimented FFA images were collected by KAWA VX-3 Ocular Fundus Digital Angiographic Processing System. The study was approved by the local medical ethics committee and each participant signed an informed consent form. With the combination of Gauss white noises with a mean value of 0 and an variance σ = 0.05, it was image decomposed by Daubechies8 Wavelet. The data was handled with the MATLAB2013 Software in the DELL Image Processing Station with a main frequency of 3.4GHz and a memory of 16GB [19-21]. Besides, the denoising algorithms of mean filter, median filter and wavelet soft-threshold were also adopted to do a denoising analysis for FFA images, and the comparison of results is shown as Fig. (**2**).

The peak signal noise ratio(PSNR) was adopted to evaluate the effects of image denoising.

(15) $$PSNR=10\log_{10}\frac{255^{2}}{\frac{1}{M\times N}\sum_{x=1}^{M}\sum_{y=1}^{N}{\left[F\left(x,y\right)-f^{\prime }\left(x,y\right)\right]}^{2}}$$

Among which, F(x,y)  is the gray value of pixel point for ideal images, $f^{\prime }\left(x,y\right)$ is the gray value of pixel point for denoised images. PSNR reflects the fidelity of noise images, and the bigger the value is, the protection for details is better. Because of the randomness of noise-adding for images, for every methods, the calculation was repeated ten times, and the mean PNSR of whose results was adopted, shown as Table **1**.

As is shown in experimental result, the algorithm adopted in this paper considered the energy sustainability and aggregation of wavelet coefficients among and inside the scales, which is better than the mean filter and median filter of single scale in denoising medical images. Besides, since the interrelationship among pixel points of images was taken onto consideration, its performance is better than wavelet soft-threshold, which can maintain the information details of FFA images to the largest extent and assist the clinical diagnosis of doctors better.

## Figures and Tables

**Fig. (1):** Wavelet coefficients arrangement.

**Fig. (2):** HMT model.

**Fig. (3):** Performance comparison of various denoising methods.

The article "The Application of Wavelet-Domain Hidden Markov Tree Model in Diabetic Retinal Image Denoising" was published in 2015. Journal: Open Biomed Eng J.

**Table 1.** PSNR values of image denoised by various methods.

WGN σ		0.05	0.1
Noisy image		20.1583	13.9004
The traditional method	Mean filter	23.0227	19.5613
	Median filter	25.4856	22.4482
The wavelet method	Soft threshold	25.8712	21.9881
	HMT	28.9977	25.8841
